# Clinical Efficacy and Safety Evaluation of Calcitriol Combined with Bisphosphonates in the Therapy of Postmenopausal Osteoporosis: Based on a Retrospective Cohort Study

This article has been retracted.

**DOI:** 10.1155/2022/2711938

**Published:** 2022-10-04

**Authors:** Weibing Jing, Yankun Dai, Jinxin Zhu, Suqin Deng

**Affiliations:** ^1^The People's Hospital of Danyang, Affiliated Danyang Hospital of Nantong University, Danyang 212300, China; ^2^Hand And Foot Surgery, The Affiliated Huai'an Hospital of Xuzhou Medical University and The Second People's Hospital of Huai'an, Huai'an 223002, China; ^3^Science and Education, Lianshui County People's Hospital, Lianshui 223400, China; ^4^Department of Pharmacy, People's Hospital of Hongze District, Huai'an 223100, China

## Abstract

A retrospective cohort study to explore the clinical efficacy and safety evaluation of calcitriol combined with bisphosphonates in the therapy of postmenopausal osteoporosis is conducted. The postmenopausal osteoporosis sufferers admitted to our hospital from January 2020 to June 2021 are retrospectively collected and divided into a contrast set and a study set, with 60 cases in each set. For the contrast set, all sufferers are treated with bisphosphonates. For the study set, on the basis of the therapy drugs in the contrast set, they are treated with calcitriol capsules. Firstly, the curative effects, bone mineral density standards, and bone metabolism standards of the two sets are contrasted; then, the lumbar spine bone mineral density, VAS score, and quality of life between the two sets of sufferers before therapy and 1 year after therapy are contrasted, and the correlation between bone mineral density and VAS and quality of life of the sufferers is analyzed. Lastly, the readmission situation between the two sets at one year is contrasted. The experimental results show that for postmenopausal women with osteoporosis, calcitriol combined with bisphosphonate therapy can notoriously enhance the clinical therapy effect of sufferers, with low adverse reactions, and can effectively enhance the bone mineral density and bone density of sufferers.

## 1. Introduction

With the continuous enhancement of living standards, the prevalence of clinical osteoporosis is increasing year by year. Osteoporosis, is caused by endocrine, metabolic, and systemic ailments. The rate is very high, which seriously affects the health and daily life of sufferers. Osteoporosis is a metabolic ailment characterized by low bone mass, destruction of bone tissue microarchitecture, and subjoined susceptibility to fractures due to subjoined bone fragility [1, 2]. In addition, an important cause of osteoporosis is the development of menopause, which is caused by the severe lack of estrogen in postmenopausal women leading to bone mineral loss and subjoined bone fragility, leading to osteoporosis, fractures, and serious consequences for sufferers. The quality of life of sufferers is seriously affected [3].

Calcitriol is currently the most commonly used drug for the clinical therapy of osteoporosis. It is the main drug for clinical therapy and has achieved specific therapeutic effects. According to clinical studies, the combination of calcitriol and bisphosphonates is safe, and it has contributed to the prognosis of the ailment [4]. Bisphosphonates are similar to pyrophosphates, and when they are used in combination with bone mineralization matrix, they can reduce bone resorption, increase bone mass, increase bone density, and are widely used in clinical practice. In addition, calcitriol can also stimulate the activity of original osteoclasts, promote the formation of new osteoclasts, and promote bone resorption [5]. This paper analyzes and discusses the efficacy and safety of calcitriol combined with bisphosphonates in the therapy of osteoporotic ailments.

The rest of this paper is organized as follows: Section 2 discusses related work, followed by sufferers' information and therapy methods designed in Section 3.  Section 4 shows the experimental results and analysis, and Section 5 summarizes the result of theoretical and empirical analysis and puts forward the direction of the future research.

## 2. Related Work

Osteoporosis is a metabolic bone ailment characterized by lessened bone strength and bone loss caused by multiple causes, which is particularly common in clinical practice. According to its etiology, it can be divided into idiopathic and secondary. After the onset, symptoms such as low back pain and fractures often occur, which not only threaten the health of sufferers but also affect daily life and work. Therefore, clinical attention should be paid to the therapy of osteoporosis, which is an effective therapy method to effectively enhance bone density, relieve symptoms, reduce side effects, and enhance the quality of life of sufferers [6, 7]. At this stage, the clinical therapy of this ailment is mainly drug therapy, and there are many types. Different drugs have different mechanisms of action. According to the different mechanisms of action of commonly used drugs, they can be divided into basic drugs, bone promoters, and bone inhibitors [8]. This study found that the total effective rate of therapy in the study set was 91. 67%, which was notoriously higher than that in the contrast set for 55.00%. The main reason for the decomposition was that bisphosphonates were more effective than other conventional drugs in the therapy of osteoporosis and could effectively promote the prognosis of the ailment. Calcitriol has the functions of fast absorption, strong affinity, few adverse reactions, and relatively long retention time of bones on human bones, thereby promoting the increase of bone density. These drugs mainly act on broken bones, effectively inhibit the activation of osteoclasts, have an extensive effect on the activation and final formation of osteoclasts, and promote the apoptosis of osteoclasts. It is relatively safe and effective in the therapy of hypercalcemia caused by inflammation, osteoporosis, and tumor bone metastasis [9, 10].

BALP is an active protease synthesized and secreted by osteoblasts, which plays an important role in the mineralization of osteoblasts and is also a marker of osteoblast maturation and differentiation [11]. Studies have shown that the decrease of serum BALP standard in sufferers with osteoporotic vertebral compression fractures will affect the bone mineral density of sufferers. PINP is the decomposition product of procollagen fibers synthesized and released by osteoblasts and is a more specific and sensitive indicator of bone formation [12]. When bone necrosis occurs, osteoclasts will stimulate osteoblasts to synthesize PINP to resist bone destruction, resulting in a compensatory increase in PINP. BGP is a noncollagen protein, which can promote the conversion of amorphous calcium phosphate to hydroxyapatite and enhance bone loss. Strength, a marker reflecting bone formation function, and lessened BGP affect the modification and reconstruction of the femur [13]. This study found that after therapy, the bone mineral density and bone metabolism in different parts of the two sets were notoriously subjoined, and the bone mineral density in the study set was notoriously higher than that in the contrast set. After therapy, the bone metabolism in both sets was notoriously subjoined, and the study set was notoriously higher. The standard of bone metabolism in the contrast set was higher than that of the contrast set (*P* < 0.05). Calcitriol is an important metabolite of vitamin D3, which can effectively promote the active absorption and utilization of calcium, phosphorus, and other minerals in the human intestine; accelerate bone metabolism; promote bone calcification; enhance bone density; and relieve bone pain symptoms. Bone metabolism is a process in which osteoclasts and osteoblasts work together to complete bone resorption and bone formation. When osteoclast function is more than osteoblasts, it will lead to bone loss and loss of bone mass, leading to osteoporosis. This process is well reflected [14]. After therapy, the VAS scores of the two sets were notoriously lessened, and the VAS scores of the study set were notoriously higher than those of the contrast set. After therapy, the quality of life scores of the two sets were subjoined, and in contrast with the contrast set, the quality of life of the study set was notoriously higher than that of the contrast set (*P* < 0.05), the main reason for the decomposition is that calcitriol plays a key role in regulating calcium balance and has a good stimulating effect on the activity of osteoblasts in bones, thus providing a good pharmacological effect for the therapy of osteoporosis. At the same time, the drug can be rapidly absorbed and reach the peak plasma concentration within 3 to 6 hours, so the onset of action is faster [15]. Zoledronic acid belongs to the class of bisphosphonates and is mostly used for the therapy of hypercalcemia and osteoporosis, which is especially obvious. It can effectively reduce the incidence of fractures, bone ailment, and bone pain and at the same time reduce symptoms, help prevent osteitis deformans, and has important value for the prognosis of the ailment [16, 17].

In addition, this study also found that there was an extensive negative correlation between bone mineral density and VAS score and an extensive positive correlation with quality of life. In June 2022, the readmission of 120 sufferers in the past year was collected, and it was found that 11 of the 35 cases were readmitted to the hospital, which was notoriously subjoined than the contrast set of 35 cases of readmission (*P* < 0.05). The main cause of postmenopausal osteoporosis in women was the decrease of estrogen standard, the weakened inhibitory effect on osteoclasts, and the osteoclast bone subjoined resorption capacity, while bone formation is insufficient to compensate for bone resorption, resulting in lessened bone mass, severe bone destruction, and weakened bone strength. Antiosteoporosis drugs can increase bone mineral density and reduce the risk of fragility fractures and are currently the main means of treating postmenopausal osteoporosis [18]. According to the mechanism of action, antiosteoporosis drugs can be divided into bone resorption inhibitors, bone formation promoters, drugs with other mechanisms, and traditional Chinese medicine. Combining antiosteoporosis drugs with the same mechanism or different mechanisms to achieve better therapeutic effect is also the current examination hot spot. Calcitriol belongs to active vitamin D and its analogs, which can increase the absorption of calcium and phosphorus in the gastrointestinal and renal tubules of sufferers. It has a good effect on improving the prognosis of sufferers [19].

## 3. Sufferers' Information and Therapy Methods

### 3.1. Sufferers' Information

The postmenopausal osteoporosis sufferers admitted to our hospital from January 2020 to June 2021 are retrospectively collected and divided into a contrast set and a study set, 60 cases in each set, according to the actual drug use of the sufferers. All sufferers meet the relevant diagnostic criteria of the “Recommended Diagnostic Criteria for Osteoporosis in China” [20]. They do not take drugs that affect bone metabolism in the recent 6 months. Sufferers and their families gave informed consent to the content of this study. The contents are as follows: those with a history of gynecological surgery in the past; those with immune system ailments such as rheumatoid arthritis and systemic lupus erythematosus; those with metabolic ailments such as hyperthyroidism, hypothyroidism, and diabetes; those who are allergic to the drugs in this study; those with severe liver ailment and renal dysfunction; incomplete data; and unable to determine the efficacy. The age of the study set is 51-64 years, with an average of 57.13 ± 5.35 years. The ailment duration is 3-16 years, with an average of 8.82 ± 5.93 years. The menopause time is 1-6 years, with an average of 3.68 ± 1.35 years. In the contrast set, the age ranged from 51 to 63 years, with an average of 57.3 ± 5.18 years. The ailment duration is from 4 to 15 years, with an average of 8.61 ± 5.16 years. The time of menopause is 1 to 5 years, with an average of 3.88 ± 1.23 years. There is no extensive disparity in general data between the two sets (*P* > 0.05), and the sets could be contrasted and analyzed. This study is reviewed and approved by the Medical Ethics Committee of our hospital. All sufferers included in the study signed the informed consent form. The therapy methods and detection methods used in this study are all known safe methods in the clinic. The general information and clinical data collected in this study are only used for examination decomposition, not for examination purposes. If you have any discomfort during the therapy, please inform your doctor in charge in time to decide the next therapy plan. During the entire therapy and observation period, please inform the doctor of the changes in your condition in time, and do not use any therapy without permission during the therapy Please inform your physician about other medicines and other therapy for this ailment.

### 3.2. Examination Methods

The examination methods of the contrast set are as follows: all sufferers are treated with bisphosphonates. First, 1 g dose of calcium gluconate injection is mixed with 500 ml of 0.9% sodium chloride injection, and intravenous drip is performed, and then, the sufferers are treated with bisphosphonates. 100 ml of zoledronic acid was intravenously infused at a constant speed, and the infusion time should be more than 5 mg in 1 minute.

The examination methods of the study set are as follows: on the basis of the therapy drugs in the contrast set, they are treated with calcitriol capsules, and 0.25 *μ*g of this product is administered orally once a day when getting up in the morning. The effect is observed after 1 month of continuous medication.

### 3.3. Efficacy Evaluation Criteria

There are three efficacy evaluation criteria as follows: (1) extensive effect: after therapy, the low back pain and accompanying symptoms disappeared or enhanced notoriously, and the bone mineral density subjoined by ≥0.06 g/cm^2^; (2) effective: after therapy, the low back pain and accompanying symptoms are enhanced, and the bone mineral density value subjoined <0.06 g/cm^2^; and (3) ineffective: after therapy, the low back pain and accompanying symptoms did not enhance or even worsened, and the bone mineral density did not increase or continued to decrease.

### 3.4. Observation Indicators

There are seven observation indicators as follows:

1. Contrast of BMD standards in different parts of the two sets of sufferers before and after therapy: dual-energy X-ray absorptiometry (DEXA) is used to detect the BMD of the lumbar spine, femoral neck, and femoral trochanter before and after therapy in the two sets of sufferers
2. Contrast of bone metabolism standards in the two sets before and after therapy: Enzyme-linked Immunosorbent Assay (ELISA) is used to detect Bone Alkaline Phosphatase (BALP), osteocalcin (BGP), and Bone-type Alkaline Phosphatase (BALP) in the two sets before and after therapy. Procollagen I N-Terminal Propeptide (PINP).
3. Measure the average lumbar bone mineral density of sufferers before therapy and 1 year after therapy, which is still done by DEXA (dual-energy X-ray absorptiometry)
4. Contrast of pain Visual Analog Scale (VAS) scores between the two sets of sufferers before and after therapy: the VAS score is used to evaluate the degree of bone pain in the two sets before and after therapy, in which 0 point indicates no pain symptoms, 10 points indicate severe pain, unbearable; the higher the score, the more severe the pain
5. Compare the quality of life between the two sets after one year of therapy
6. To analyze the correlation between bone mineral density and VAS and quality of life of sufferers
7. The one-year readmission of the two sets is contrasted. In June 2022, the readmission of 120 sufferers in the past year are collected. Calculate their cumulative readmission rate

### 3.5. Statistical Methods

First, create an excel sheet, organize the data required for this study according to sets, open SPSS 26.0, and enter the data into decomposition, respectively. For the measurement data, normality and variance homogeneity tests are performed on them, all of which are normally distributed data, indicating that the test methods are$\bar{x}\pm s$and*t*, respectively. Measurement data representation and test methods are *n* (%) and *χ*^2^, respectively. Correlation is analyzed by Pearson. When *P* < 0.05, it is considered that there is a disparity between the data. The disparity is statistically extensive.

## 4. Experimental Results

### 4.1. Contrast of Curative Effects between the Two Sets after Therapy

Table 1 shows the contrast of curative effects between the two sets after therapy. It can be seen from Table 1 that the total effective rate of the study set is 91. 67%, which is notoriously higher than that of the contrast set for 55.00%, and the disparity is statistically extensive (*P* < 0.05) after therapy.

### 4.2. Contrast of Bone Mineral Density Standards in Different Parts of the Two Sets before and after Therapy

Table 2 shows the contrast of bone mineral density in different parts before and after therapy in two sets of sufferers. In Table 2, ∗ indicates that contrast with before therapy in this set, *P* < 0.05. It can be seen from Table 2 that there is no extensive disparity in bone mineral density in different parts of the two sets, and the standards are notoriously subjoined (*P* > 0.05) before therapy. After therapy, the bone mineral density in different parts of the two sets is notoriously subjoined, and the bone mineral density in the study set is notoriously higher than that in the contrast set (*P* < 0.05).

### 4.3. Contrast of Bone Metabolism Standards in the Two Sets before and after Therapy

Table 3 shows the contrast of bone metabolism standards in the two sets of sufferers before and after therapy. In Table 3, ∗ indicates that contrast with before therapy in this set, *P* < 0.05. It can be seen from Table 3 that there is no extensive disparity in the standard of bone metabolism between the two sets, and the standards are notoriously subjoined (*P* > 0.05) before therapy. After therapy, the standards of bone metabolism in both sets are notoriously subjoined, and the standard of bone metabolism in the study set is notoriously higher than that in the contrast set (*P* < 0.05).

### 4.4. Contrast of Lumbar Spine Bone Mineral Density Values before Therapy and 1 Year after Therapy between the Two Sets

Table 4 shows the lumbar vertebra bone mineral density values before therapy and 1 year after therapy in two sets. In Table 4, ∗ indicates that contrast with before therapy in this set, *P* < 0.05. It can be seen from Table 4 that there is no extensive disparity in the bone mineral density of the lumbar vertebrae between the two sets, and the standards are notoriously subjoined (*P* > 0.05) before therapy. After therapy, the BMD of the lumbar vertebrae in both sets are notoriously subjoined, and the BMD of the lumbar vertebrae in the study set is notoriously higher than that in the contrast set (*P* < 0.05).

### 4.5. Contrast of VAS Scores before and One Year after Therapy between the Two Sets

Table 5 shows the contrast of VAS scores between the two sets of sufferers before and one year after therapy. In Table 5, ∗ indicates that contrast with before therapy in this set, *P* < 0.05. It can be seen from Table 5 that there is no extensive disparity in VAS scores between the two sets, and the standards are notoriously higher (*P* > 0.05) before therapy. After therapy, the VAS scores in both sets are notoriously lessened, and the VAS scores in the study set are notoriously higher than those in the contrast set (*P* < 0.05).

### 4.6. Contrast of the Quality of Life between the Two Sets before and One Year after Therapy

Table 6 shows the contrast of quality of life between the two sets before and one year after therapy. In Table 6, ∗ indicates that contrast with before therapy in this set, *P* < 0.05. It can be seen from Table 6 that there is no extensive disparity in the quality of life between the two sets, and the standards are relatively low (*P* > 0.05) before therapy. After therapy, the quality of life scores in both sets are subjoined, and in contrast with the contrast set, the quality of life in the study set is notoriously higher (*P* < 0.05).

### 4.7. Contrast of the Incidence of Adverse Reactions between the Two Sets

During the drug therapy period, 1 case of nausea and 2 cases of vomiting occur in the contrast set and 2 cases of nausea, 2 cases of vomiting, and 1 case of drowsiness in the study set, but the symptoms are all weak, and there are no other serious adverse reactions (*P* > 0.05).

### 4.8. Decomposition of the Correlation between Bone Mineral Density and VAS and Quality of Life in Sufferers

Table 7 shows the correlation of bone mineral density with VAS and quality of life.  Figure 1 shows the correlation between bone mineral density and VAS.  Figure 2 shows the correlation between bone mineral density and quality of life. Through the above experimental results, it can be observed that the BMD, VAS, and quality of life data of sufferers before and after therapy are collected, and the first Pearson decomposition is performed. It is found that there is an extensive negative correlation between BMD and VAS score. There is an extensive positive correlation with the quality of life (both *P* < 0.05).

### 4.9. Comparing the Cumulative Rate of Readmission between the Two Sets

In June 2022, the readmissions of 120 sufferers in the past year are collected.  Figure 3 shows the contrast of the cumulative rate of readmission between the two sets. It can be seen from Figure 3 that there are 11 readmissions in the study set, which is notoriously subjoined than the 35 readmissions in the contrast set (*P* < 0.05).

## 5. Conclusion

A retrospective cohort study to explore the clinical efficacy and safety evaluation of calcitriol combined with bisphosphonates in the therapy of postmenopausal osteoporosis is conducted. For postmenopausal women with osteoporosis, calcitriol combined with bisphosphonate therapy can notoriously enhance the clinical therapy effect of the sufferers, with low adverse reactions, and can effectively enhance the bone mineral density and bone metabolism of the sufferers. The prognosis of sufferers is worthy of clinical application.

## Figures and Tables

**Figure 1:** Correlation between bone mineral density and VAS.

**Figure 2:** Correlation between bone mineral density and quality of life.

**Figure 3:** Contrast of the cumulative rate of readmission between the two sets.

**Table 1:** Contrast of curative effects between the two sets after therapy.

Set	Effective	Valid	Invalid	Total efficiency
Contrast set (*n* = 60)	15	18	27	33 (55.00)
Study set (*n* = 60)	35	20	5	55 (91.67)
*χ* ^2^				26.625
*P*				<0.001

**Table 2:** Contrast of bone mineral density in different parts before and after therapy in two sets of sufferers (g/cm^2^).

Set	Lumbar position		Femoral neck		Femoral tuberosity	
	Before therapy	After therapy	Before therapy	After therapy	Before therapy	After therapy
Study set (*n* = 60)	0.59 ± 0.11	0.78 ± 0.07^∗^	0.65 ± 0.15	0.82 ± 0.10^∗^	0.71 ± 0.07	0.88 ± 0.09^∗^
Contrast set (*n* = 60)	0.58 ± 0.10	0.70 ± 0.08^∗^	0.64 ± 0.13	0.75 ± 0.09^∗^	0.72 ± 0.08	0.81 ± 0.08^∗^
*t*	0.521	5.829	0.390	4.030	-0.729	4.503
*P*	0.603	<0.001	0.697	<0.001	0.428	<0.001

**Table 3:** Contrast of bone metabolism standards in the two sets of sufferers before and after therapy.

Set	BALP (U/l)		BGP (*μ*g/ml)	
	Before therapy	After therapy	Before therapy	After therapy
Study set (*n* = 60)	79.78 ± 10.36	92.54 ± 10.59^∗^	1.44 ± 0.37	2.84 ± 0.52^∗^
Contrast set (*n* = 60)	78.96 ± 10.25	83.7 ± 11.25^∗^	1.43 ± 0.36	2.18 ± 0.41^∗^
*t*	0.436	4.432	0.150	7.720
*P*	0.664	<0.001	0.881	<0.001

**Table 4:** Lumbar vertebra bone mineral density values before therapy and 1 year after therapy in two sets.

Set	Bone density (g/cm^2^)	
	Before therapy	1 year after therapy
Study set (*n* = 60)	0.65 ± 0.11	0.81 ± 0.08^∗^
Contrast set (*n* = 60)	0.64 ± 0.13	0.76 ± 0.07^∗^
*t*	0.455	3.643
*P*	0.650	<0.001

**Table 5:** Contrast of VAS scores between the two sets of sufferers before and one year after therapy.

Set	VAS (score)	
	Before therapy	1 year after therapy
Study set (*n* = 60)	7.45 ± 1.13	2.23 ± 0.67^∗^
Contrast set (*n* = 60)	7.40 ± 1.15	4.72 ± 1.57^∗^
*t*	0.240	-11.299
*P*	0.811	<0.001

**Table 6:** Contrast of quality of life between the two sets before and one year after therapy.

Set	Quality of life (score)	
	Before therapy	1 year after therapy
Study set (*n* = 60)	64.48 ± 8.25	85.31 ± 4.17^∗^
Contrast set (*n* = 60)	67.15 ± 7.93	77.67 ± 5.26^∗^
*t*	-1.807	8.816
*P*	0.073	<0.001

**Table 7:** Correlation of bone mineral density with VAS and quality of life.

	Bone density	
	*r*	*P*
VAS	-0.759	<0.001
Quality of life	0.826	<0.001

## Data Availability

The simulation experiment data used to support the findings of this study are available from the corresponding author upon request.
